# Intracytoplasmic Sperm Injection Improves Normal Fertilization Rate and Clinical Pregnancy Rate in Male Infertility

**DOI:** 10.1155/2022/1522636

**Published:** 2022-07-31

**Authors:** Jiqun Xu, Yi Yu, Mingyue Xue, Xiangyang Lv

**Affiliations:** Center for Integrative Medicine Reproduction and Genetics, Affiliated Hospital of Shandong University of Traditional Chinese Medicine, Jinan, China

## Abstract

The purpose of this study was to investigate the effect of intracytoplasmic sperm injection (ICSI) on the normal fertilization rate of oocytes and the clinical pregnancy rate of cycles in male infertility. Eighty cases of male infertility patients attending our hospital from March 2020 to March 2021 were selected and divided into observation group and control group using the random number table method, with 40 cases in each group. The control group was treated with in vitro fertilization (IVF), and the observation group was treated with ICSI. The normal fertilization rate of oocytes and the clinical pregnancy rate of the cycle were compared between the two groups, and the adverse pregnancy outcome and obstetric and perinatal complications were compared between the two groups The rate of normal fertilization and clinical pregnancy in the cycle was higher in the observation group (*P* < 0.05). The differences were not statistically significant (*P* > 0.05) when comparing adverse pregnancy outcomes between the two groups. The difference was not statistically significant (*P* > 0.05) when comparing obstetrics (5.41%, 10.34%) and perinatal complications (8.33%, 14.81%) between the two groups. ICSI in male infertility is significantly effective in improving the rate of normal oocyte fertilization and the clinical pregnancy rate of the cycle. It also has a low impact on adverse pregnancy outcomes and obstetric and perinatal complications and has a high safety profile.

## 1. Introduction

Male infertility is caused by male factors, and the disease has become a common clinical condition. Its prevalence is about 10%, with male factors alone accounting for about 30%. The incidence of male infertility at fertile age in China is on the rise [1]. One study reported an infertility rate of 45% in 117,979 men, with semen reports showing oligospermia (22%), weak sperm (11%), and azoospermia (12%) as major factors [2]. Male infertility not only affects reproductive health and the birth rate of newborns in society but also affects the psychological health of patients and causes depression, anxiety, and obsessive-compulsive pathology, increasing the psychological burden and reducing the quality of life of patients [3, 4]. Therefore, it is important to study techniques for the prevention and treatment of male infertility. Most patients are treated with assisted reproductive techniques. Among these techniques, intracytoplasmic single sperm injection (ICSI) is a common clinical assisted reproduction technique with the advantage of being independent of sperm count and morphology and having a high fertilization rate [5, 6]. In recent years, multicental randomised controlled trials have been conducted overseas to analyze the effects of ICSI on offspring compared with traditional in vitro fertilization techniques [7]. However, clinical studies in China have mainly focused on the effects of ICSI in male infertility with different sperm sources, while the effects of ICSI and traditional in vitro fertilization (IVF) on offspring have not been reported, and further studies are still needed. Based on this, this study will analyze the effects of different techniques of ICSI and traditional in vitro fertilization in male infertility. The purpose of this study is to determine the effect of ICSI on the normal fertilization rate of oocytes and the clinical pregnancy rate of cycles, and to further provide more ideal assisted reproductive technology for patients.

## 2. Patients and Methods

### 2.1. Patients

Eighty male infertility patients who visited our hospital from March 2020 to March 2021 were selected and randomly divided into observation group (*n* = 40) and control group (*n* = 40). In the observation group, the male age was 24–41 years (31.27 ± 2.24) years, the female age was 23–39 years (30.25 ± 2.18) years; the duration of infertility was 0.5–17 years (4.16 ± 1.25) years. In the control group, the age of the man was 22–39 years (31.14 ± 2.35) years and the age of the woman was 22–37 years (30.29 ± 2.12) years; the duration of infertility was 0.5–16 years (4.17 ± 1.26) years. There was no significant difference in the general data between the two groups (*P* > 0.05).

All patients were referred to the relevant diagnostic criteria [8]: couples who had regular sexual intercourse for 1 year and were not using contraception; patients were confirmed by semen analysis and other laboratory and imaging techniques to have severe oligo-(weak) sperm nonliquefaction, obstructive azoospermia and other types. Inclusion criteria were as follows: (1) patients were eligible for male infertility; (2) patients were planning to undergo their first IVF or ICSI cycle; (3) patients signed an informed consent form before the treatment. Exclusion criteria were as follows: (1) patients with comorbid psychiatric disorders, depression, liver and kidney dysfunction, cardiovascular disease, etc.; (2) patients with contraindications to IVF or ICSI; (3) patients with poor fertilization (≤25%) in the previous cycle; (4) patients who did not cooperate with the follow-up. The study protocol was in accordance with the Helsinki Declaration and had been approved by our ethics committee.

### 2.2. Method

All the couples in the study received short-acting gonadotropin-releasing hormone (GnRH) antagonist regimen. On the second day, they began to inject gonadotropin with a dose of 0.5–1.0 mg for 14 days. After reaching the standard, they began to promote ovulation. Recombinant follicle-stimulating hormone (rFSH) was given and the follicular development was monitored by transvaginal B-ultrasound. When there were two follicles with diameters ≥18 mm, 250 *μ*g of human chorionic gonadotrophin *p* (p-HCG) was subcutaneously injected. After 34–36 h, the puncture and ovulation were performed under transvaginal B-ultrasound and put into the culture medium for 6 h in a suitable state (37 °C, 6% CO_2_). Fresh ejaculatory semen samples were obtained by masturbation after 2–7 days of oocyte extraction, and the samples were prepared by density gradient centrifugation. At the same time, the sperm morphology was observed under a microscope.

The control group underwent IVF treatment, completed conventional treatment, and observed the presence of the first diode. The observation group was treated with ICSI, and the operation was as follows: the culture medium containing hyaluronidase was added to the oocyte preparation to digest and remove the granulosa cells around the egg, and the preparation for microinjection was completed. We transferred the eggs of granulosa cells to the microdroplets in the operating dish, each drop with a second meiosis metaphase egg; the egg was fixed with an egg needle to keep it in the body position at 12'O clock. At the same time, the normal sperm was selected to brake the sperm with a microinjection needle, and the sperm was inhaled with a tail-to-head injection needle and vertically penetrated the cytoplasm from 3'O clock. After ensuring the rupture of the membrane, sperm was injected into the cytoplasm together; at the same time, the microinjection needle was removed and the fixed needle was loosened to release the eggs. After all the eggs were injected, they were transferred to a Petri dish containing embryonic culture medium and cultured at suitable conditions (37°C, 6% CO_2_) for 6 h. After 16–18 h of injection, the inverted microscope was used to examine the fertilization of eggs under 200-fold parameters. The normal fertilization state showed the presence of dikaryocyte and the discharge of the second polar body. 72∼78 h after oocyte retrieval, the cleavage of embryos was carefully observed, and the high-quality embryos were screened for vaginal implantation into the uterine cavity. At the same time, 1–3 embryos were transplanted per cycle according to the age of the female, and the remaining high-quality embryos were cryopreserved; patients with inferior embryos were informed and their blastocysts were cultured or discarded with their consent. After 14 days of transplantation, laboratory indexes such as urine and blood human chorionic gonadotropin were monitored, and biochemical pregnancy was positive. After 30 days of transplantation, B-ultrasound examination was performed, showing that the gestational sac and cardiac catheterization were clinically pregnant.

### 2.3. Outcome Measures

The normal fertilization rate of oocytes and cycle clinical pregnancy rate were compared between the two groups: normal fertilization rate = number of normal fertilizations/number of oocytes retrieved 100% (fertilization is defined as 2 PN fertilized eggs); cycle clinical pregnancy rate = number of clinical pregnancies/number of transfer cycles 100%. Adverse pregnancy outcomes were compared between the two groups: continuous follow-up until adverse outcomes were produced or 6 weeks after delivery, including miscarriage (termination of pregnancy before 28 weeks), preterm delivery (birth between 28 and 37 weeks of gestation), perinatal mortality (death in late pregnancy, delivery, or within 7 days after birth), and neonatal mortality (death of live births within 28 days after birth). Obstetric and perinatal complications were compared between the two groups: obstetric complications included gestational diabetes and hypertension, and perinatal complications included congenital abnormalities and macrosomia after 6 weeks of continuous follow-up until delivery.

### 2.4. Statistical Analysis

Statistical Product and Service Solutions (SPSS) 23.0 (SPSS Inc., Chicago, IL, USA) was applied for statistical analysis. The independent sample *t*-test was used for comparison between groups for measurement data obeying normal distribution, and the independent sample *t*-test was used for comparison within groups, all expressed as (*x̅* ± *s*). The count data were tested by *χ*^2^ and expressed as rate (%), and *P* < 0.05 indicates a statistical difference.

## 3. Results

### 3.1. The Normal Fertilization Rate of Oocytes and Clinical Pregnancy Rate of Cycles between the Two Groups

In the observation group, 913 eggs were obtained in 90 treatment cycles, including 843 eggs in the second meiotic metaphase (MII); in the control group, 897 eggs were obtained in 90 treatment cycles, including 811 eggs in the second meiotic metaphase (MII). Fresh embryo transfer was performed in 42 cycles of clinical pregnancy in both groups. The normal fertilization rate and cycle clinical pregnancy rate in the observation group were higher than those in the control group (*P* < 0.05) (Table 1).

### 3.2. Adverse Pregnancy Outcomes between the Two Groups

There was no significant difference in adverse pregnancy outcomes (abortion (2.70%, 6.90%), premature delivery (5.41%, 10.34%), perinatal mortality (8.11%, 6.90%), and neonatal mortality (5.41%, 3.45%)) between the two groups (*P* > 0.05) (Table 2).

### 3.3. Obstetric and Perinatal Complications between the Two Groups

There was no significant difference in obstetric (5.41%, 10.34%) and perinatal complications between the two groups (8.33%, 14.81%) (*P* > 0.05) (Table 3).

## 4. Discussion

Male infertility has become a public health problem of global concern. There are more and more clinical studies on the etiology and pathogenesis of this disease. Related research reports [9] show that overweight, chronic diseases, living habits and genetic factors are all risk factors for male infertility. Overweight factors mainly reduce male fertility by influencing sexual development, endocrine disorders, semen quality and psychology. Chronic diseases such as hypertension and diabetes mainly reduce male fertility by influencing hormone levels, reducing gonadal function and sexual function. Living habits include staying up late, smoking, drinking, and lack of exercise, which mainly reduce fertility by influencing hormone secretion and reducing sperm activity. Most genetic factors are genetic defects such as Kirsch syndrome and 47XYY syndrome, which lead to disorder or abnormality in spermatogenesis. With the in-depth study of the pathogenesis of male infertility, it is more scientific and accurate to formulate individualized treatment strategies. It is clinically believed that the formation of this disease is mainly related to the oxidative stress mechanism that affects sperm capacitation, acrosome reaction and tissue damage. Abnormal signaling pathways such as amino acids and fatty acid derivatives lead to dysfunction of sperm function [10, 11].

With the development and maturity of microsurgical techniques, the application of this technique in assisted reproductive techniques has also become increasingly widespread [12]. The ICSI operation process includes the in vitro culture process of gametes and embryos, and the technique of selecting high-quality individual sperm with the help of microinjector operating system and mechanically injecting their sperm into oocytes to complete the fertilization process [13–15]. For patients whose sperm count is too low or morphological and functional defects lead to the inability to penetrate the zona pellucida of oocytes normally, ICSI technique can be used to obtain sperm and improve fertilization rate. However, there are clinical concerns about technology involving damage to gametes and offspring health status, and some studies suggest that this process interferes with gametogenesis, embryo development, and the environment of the pregnancy process, and exogenous substances are injected into the oocyte proton during the operation, which easily damages tissue structures such as eggs and spindles, and then has adverse effects on fertilization of gametes and subsequent embryo differentiation and development [16, 17]. Therefore, it is necessary to conduct an in-depth study of the effects of ICSI technology on offspring. The results of this study showed that the normal fertilization rate and cycle clinical pregnancy rate in the observation group were higher than those in the control group (*P* < 0.05). The normal fertilization rate and cycle clinical pregnancy rate in the observation group were higher than those in the control group (*P* < 0.05). There was no significant difference in adverse pregnancy outcomes (abortion (2.70%, 6.90%), premature delivery (5.41%, 10.34%), perinatal mortality (8.11%, 6.90%), and neonatal mortality (5.41%, 3.45%)) between the two groups (*P* > 0.05). There was no significant difference in obstetric (5.41%, 10.34%) and perinatal complications between the two groups (8.33%, 14.81%) (*P* > 0.05). These results indicate that ICSI technique has a good therapeutic effect, and has no significant effect on live birth rate, obstetric and perinatal complications. The limitations of the article was that the article was a single-centre study and there may be some bias in the selection of patients. Therefore, a multicentral, randomised, double-blind study was needed to further confirm the findings of this study.

## 5. Conclusion

ICSI is effective in male infertility and can improve the normal fertilization rate of oocytes and the clinical pregnancy rate of cycles, with little effect on adverse pregnancy outcomes and obstetric and perinatal complications and has high safety.

## Figures and Tables

**Table 1:** Comparison of normal oocyte fertilization rate and cycle clinical pregnancy rate between the two groups (*n* = 40, (%)).

Group	Normal fertilization rate	Interval clinical pregnancy rate
Observation group	88.02 (742/843)	88.10 (37/42)
Control group	83.72 (679/811)	69.05 (29/42)
Χ^2^	6.301	4.525
*P* value	0.012	0.033

**Table 2:** Comparison of adverse pregnancy outcomes between the two groups (*n*, (%)).

Group	Number of subjects	Abortion	Premature	Perinatal mortality	Neonatal mortality
Observation group	37	1 (2.70)	2 (5.41)	3 (8.11)	2 (5.41)
Control group	29	2 (6.90)	3 (10.34)	2 (6.90)	1 (3.45)
Χ^2^	—	0.659	0.567	0.034	0.144
*P* value	—	0.417	0.452	0.854	0.705

**Table 3:** Comparison of obstetrical and perinatal complications between the two groups (*n*, (%)).

Group	Gestational diabetes	Gestational hypertension	Obstetric complications	Congenital anomaly	Macrosomia	Perinatal complications
Observation group	2.70 (1/37)	2.70 (1/37)	5.41 (2/37)	2.78 (1/36)	5.56 (2/36)	8.33 (3/36)
Control group	3.45 (1/29)	6.90 (2/29)	10.34 (3/29)	7.41 (2/27)	7.41 (2/27)	14.81 (4/27)
Χ^2^	—	—	0567	—	—	0.656
*P* value	—	—	0.452	—	—	0.418

## Data Availability

The datasets used and analyzed during the current study are available from the corresponding author on reasonable request.

## References

[1] Guzick D. S., Overstreet J. W., Factor-Litvak P. (2001). Sperm morphology, motility, and concentration in fertile and infertile men. *New England Journal of Medicine*.

[2] Mehra B. L., Skandhan K. P., Prasad B. S., Pawankumar G., Singh G., Jaya V. (2018). Male infertility rate: a retrospective study. *Urologia Journal*.

[3] Kasman A. M., Zhang C. A., Luke B., Eisenberg M. L. (2020). Association between infertility and mental health of offspring in the United States: a population based cohort study. *Human Fertility*.

[4] Massarotti C., Gentile G., Ferreccio C., Scaruffi P., Remorgida V., Anserini P. (2019). Impact of infertility and infertility treatments on quality of life and levels of anxiety and depression in women undergoing in vitro fertilization. *Gynecological Endocrinology*.

[5] Esteves S. C., Roque M., Bedoschi G., Haahr T., Humaidan P. (2018). Intracytoplasmic sperm injection for male infertility and consequences for offspring. *Nature Reviews Urology*.

[6] Meschede D., Lemcke B., Exeler J. R. (1998). Chromosome abnormalities in 447 couples undergoing intracytoplasmic sperm injection--prevalence, types, sex distribution and reproductive relevance. *Human Reproduction*.

[7] Zheng D., Zeng L., Yang R. (2019). Intracytoplasmic sperm injection (ICSI) versus conventional in vitro fertilisation (IVF) in couples with non-severe male infertility (NSMI-ICSI): protocol for a multicentre randomised controlled trial. *Bmj Open*.

[8] Schlegel P. N., Sigman M., Collura B. (2021). Diagnosis and treatment of infertility in men: AUA/ASRM guideline part II. *Journal of Urology*.

[9] Winters B. R., Walsh T. J. (2014). The epidemiology of male infertility. *Urologic Clinics of North America*.

[10] Liu L., Wang H., Tian M. (2017). Phthalate metabolites related to infertile biomarkers and infertility in Chinese men. *Environmental Pollution*.

[11] Gunes S., Esteves S. C. (2021). Role of genetics and epigenetics in male infertility. *Andrologia*.

[12] Mcloughlin M. G. (1980). The role of microsurgery in male infertility. *Clinical Obstetrics and Gynecology*.

[13] Giacobbe M., Conatti M., Gomes A., Bonetti T. C., Monteleone P. A. (2022). Effectivity of conventional in vitro fertilization (IVF) and intracytoplasmic sperm injection (ICSI) when male factor is absent: a perspective point of view. *JBRA Assisted Reproduction*.

[14] Zorn B., Vidmar G., Meden-Vrtovec H. (2003). Seminal reactive oxygen species as predictors of fertilization, embryo quality and pregnancy rates after conventional in vitro fertilization and intracytoplasmic sperm injection. *International Journal of Andrology*.

[15] Gordts S., Rombauts L., Roziers P. (1998). Intracytoplasmic sperm injection in the treatment of male subfertility. *European Journal of Obstetrics & Gynecology and Reproductive Biology*.

[16] Nariyoshi S., Nakano K., Sukegawa G., Sho T., Tsuji Y. (2020). Ultrasonographically determined size of seminiferous tubules predicts sperm retrieval by microdissection testicular sperm extraction in men with nonobstructive azoospermia. *Fertility and Sterility*.

[17] Berntsen S., Nøhr B., Grøndahl M. L. (2021). In vitro fertilisation (IVF) versus intracytoplasmic sperm injection (ICSI) in patients without severe male factor infertility: study protocol for the randomised, controlled, multicentre trial INVICSI. *Bmj Open*.

